This article has been retracted.

# Effectiveness Analysis of English Newspaper Reading Teaching Based on Deep Learning from the Perspective of Online and Offline Hybrid Teaching

**DOI:** 10.1155/2022/4065527

**Published:** 2022-07-18

**Authors:** Zheng Zeng, Xi Wang

**Affiliations:** School of Foreign Languages and International Education, Chengdu Technological University, Chengdu, 611730 Sichuan, China

## Abstract

In recent years, China's higher education has developed rapidly, and the overall English proficiency of college students has improved significantly. In order to improve the English proficiency of students in higher education, English newspaper reading courses are offered, many of which are elective courses. Reading English newspapers in English can help college students improve their overall English proficiency and benefit them in their future lives. Reading English newspapers can improve students' English in many ways as part of college English teaching activities. For example, it helps students to accumulate common and authentic words and phrases, improve their English reading efficiency and level, and gain a broader perspective. This paper examines the role of English newspaper reading in college English teaching, proposes an effective analysis method of teaching English newspaper reading based on deep learning from the perspective of online and offline hybrid teaching, and tests the effectiveness of the model. Finally, the specific characteristics of English newspapers are combined to propose suggestions for improving the effectiveness of English teaching activities for college students.

## 1. Introduction

English reading teaching was first born in the United States in 1955. It mainly applies newspapers and other publications to school teaching. Its purpose is to improve students' reading ability and writing abilities [1]. At the same time, it can also help students understand and master relevant current affairs news and broaden their horizons. In China, English newspaper reading is mainly to enable English majors to improve their comprehensive ability, including improving the speed and level of reading English newspapers. At the same time, we should be familiar with and understand the writing characteristics of news articles in English-speaking countries such as the UK and the United States and be able to analyze and learn the ideas expressed in English newspapers and articles and some writing skills, so as to effectively improve the reading comprehension level of English majors [2]. In recent years, my country's higher education has developed rapidly, and the overall English level of college students has been greatly improved. Schools in some big cities have higher and higher requirements for students' English ability and have set up English newspaper reading courses for this purpose, many of which take it as an elective course. English newspaper reading can lay an important foundation for improving the comprehensive English quality of college students, so that students can benefit a lot in their future life [3].

In college English teaching, the content of English reading not only embodies important humanistic value but also has far-reaching social significance. In order to improve the comprehensive English quality of college students, we must not only emphasize the utilitarian idea of English as a tool but also pay attention to the humanistic value behind English, so that college students can deeply realize that English learning can play a great role. It has a profound impact on the cultivation of its own humanistic quality [4]. Therefore, the goal of college English teaching at this stage should not be simply to take some exams but to fully stimulate the interest and enthusiasm of learning English as a subject by reading English newspapers, so as to cultivate students' ability of independent learning and independent thinking [5]. At the same time, reading English newspapers and periodicals can also broaden students' horizons and better develop students' thinking ability and innovation abilities. After comparing English newspapers and periodicals with college school English textbooks, it can be found that English newspapers and periodicals have the advantages of internationalization, effectiveness, and practicability. Moreover, English newspapers and periodicals cover a wide range of contents, which can enable students to obtain relevant knowledge and information in various fields in the process of reading, help students understand the cultural background of different countries and regions, and enable students to more objectively understand the traditional culture and modern civilization of other countries and peoples [6]. On the other hand, to a certain extent, it can also deepen students' recognition of their own culture, which is conducive to the formation of students' correct outlook on life, and values, and lay a solid foundation for their future study, work, and life [7]. The significance and function of English newspaper reading are shown in Figure 1.

College English courses must include compulsory and elective courses. Students must take mandatory courses in order to learn fundamental English language information and develop basic English language aptitude. Simultaneously, in compulsory courses, we should promote active study habits and scientific and effective learning methods, and students should strengthen their cross-cultural communication skills [8]. Elective courses are to respect and meet the personalized characteristics of students because different students have differences in enrollment, employment, and personal interests. The content of elective courses is generally to further improve students' knowledge and skills in a small field, including English newspaper reading, English speech and debate, and primary English translation. According to relevant survey results, among college English elective courses, the most popular elective course for college students is English newspaper reading [9]. In college English teaching activities, the role of reading newspapers is very obvious. However, in the current college English teaching activities, teachers often overemphasize vocabulary, phrases, grammar, and other knowledge content in textbooks, while ignoring or not understanding the role of English newspaper reading in promoting students' English proficiency [10].

The following is a summary of the research: Section 2 contains the related work.  Section 3 discusses the design of application model of the proposed work. In Section 4 contains the experiment and analysis of the proposed concepts. Finally, the conclusion brings the paper to a finish in Section 5.

## 2. Related Work

### 2.1. Research Status of Online and Offline Hybrid Teaching

The online and offline mixed teaching paradigm is based on constructivist learning theory and the application of modern information technology to achieve the development, integration, and exploitation of a variety of teaching resources [11]. It is a revolutionary teaching approach that improves teaching efficiency and effectiveness by deeply integrating traditional offline classroom teaching content with online teaching, then maximizing the benefits of both online and traditional classroom teaching and fostering their complementarity [12]. During the practice of online and offline hybrid teaching mode, it embodies many functions, such as live recording and broadcasting, teaching interaction, teaching management, online teaching, and a course on-demand. It can effectively build a teaching platform and then organize online teaching to meet the learning needs of contemporary college students. Whether online or offline teaching, students are the main body of teaching and need to carry out various teaching activities centered on students. Therefore, students are participants in the mixed teaching mode [13]. The organization and development of teaching work should pay attention to providing students with learning support and guiding students to actively participate in the mixed teaching mode. Fully mobilize students' learning enthusiasm and initiative and promote teaching reform. The online and offline hybrid teaching mode not only organically combines the two classrooms and highlights the dominant position of students in learning but also reflects the leading role of teachers. It is a new direction of teaching reform and development in colleges and universities [14].

The characteristics of online and offline hybrid teaching are then discussed. To begin, online and offline hybrid teaching is defined as the synchronization of online and offline teaching formats in order to achieve an organic combination. Second, it must be clear that online teaching is not an auxiliary method of hybrid teaching, but the basis for the organization and implementation of teaching activities. Third, in the process of the reform of online and offline mixed teaching modes, a unified mode has not been formed [15]. However, the goal can be determined, which is to effectively improve the teaching effect and students' learning effect, and cultivate students' autonomous learning ability and good learning habits. In the process of curriculum integration teaching, we must clarify the nature of the curriculum. At present, not all the courses in colleges and universities are suitable for online and offline hybrid teaching. We should combine different courses and select the matching online teaching platform and teaching means [16]. Fourth, compared with traditional offline classroom teaching, the time and space of online and offline hybrid teaching modes are not limited, and teaching can be organized and carried out at any time or place. Therefore, the reform of online and offline mixed teaching mode is an inevitable method to break through the traditional teaching and also realizes the reconstruction of the traditional classroom. The concept of online and offline hybrid teaching is shown in Figure 2.

In fact, the online and offline mixed teaching mode reflects the most obvious characteristics, that is, it has changed the traditional teaching structure, and there are differences in the teaching structure between the online and offline mixed teaching mode and the traditional teaching [17]. Under the traditional classroom teaching mode, teachers usually assign preview tasks, and students generally understand knowledge before teaching. This preview usually lacks guidance, and even many students' preview knowledge content has nothing to do with classroom teaching. The online and offline hybrid teaching structure makes the limited classroom time more valuable. After students fully preview online, teachers do not need to waste a lot of time explaining the theoretical basis [18]. We can carry out in-depth discussions on the key and difficult knowledge, form a good classroom learning atmosphere, make full use of the limited teaching time, and promote the internalization and absorption of students' knowledge.

### 2.2. Research Status of English Reading Teaching

On the whole, domestic scholars have conducted in-depth research on English reading teaching based on the cultivation of core literacy. Although the literature has different expressions on the connotation of core literacy, most agree that focusing on core literacy is to emphasize that education should focus on people all-around and sustainable development and give full play to the “educating” function of education. Many scholars agree that reading teaching plays an irreplaceable role in cultivating the four-dimensional core literacy of English subjects, but there are many problems in cultivating students' core literacy in college English reading teaching [19]. Domestic research did not begin till recently. The majority of the research focuses on the connotation, relevance, key characteristics, and realization requirements of core literacy [20], with a particular emphasis on the advanced experience at home and abroad in recent years. The research on the interactive relationship between core literacy and education and teaching is not deep enough, the attention to the heterogeneity of the interaction between core literacy and different disciplines is not high, there is a lack of systematic research on how to achieve the educational goal of core literacy training in curriculum teaching reform, and the research on integrating core literacy into English classroom teaching, especially English Reading Teaching in college, is particularly rare. The five characteristics of English reading teaching are shown in Figure 3.

Most of the existing studies focus on the curriculum teaching practice itself from the perspective of teachers and rarely conduct in-depth research on learning subjects, teaching media, and external factors, especially the lack of relevant research on how students acquire core literacy [21]. Most of the existing studies are aimed at the teaching of reading in schools. There are few studies on how to guide students to read independently and cultivate students' core literacy after class [22]. As for how to cultivate the four-dimensional core literacy of English subjects in college English reading teaching, the existing research mainly focuses on cultivating students' thinking quality, and there are relatively few studies on the other three core literacy. Even in studies that focus on improving students' thinking skills, they tend to focus on abstract levels such as feasibility analysis, direction counseling, and strategy advice [23]. Whether they have guiding value is unknown. Therefore, looking for more practical strategies is worth further discussion. The existing research focuses on the theoretical analysis of reasons, current situation, and strategies and focuses on the experience sharing of fragmentation [24]. Although there are a small number of case studies, it has not formed a systematic and practical teaching model. Therefore, it is an important direction of future research to find an English reading classroom teaching model with universal guiding significance and based on the cultivation of students' core literacy [25]. The research on the effect of English reading teaching on the cultivation of students' core literacy is still in its infancy. Therefore, it is also an important topic of current research to construct a college English teaching evaluation system that not only conforms to the characteristics of China's education and education reform but also reflects the quality of students' core literacy training [26].

### 2.3. Research Status of Deep Learning

Deep learning belongs to machine learning and is a very important branch in the field of machine learning. Understanding the principle of machine learning will help us better understand deep learning. Machine learning is a branch of artificial intelligence. When people talk about artificial intelligence, they often cannot get around machine learning [27]. Obviously, machine learning studies how to make machines learn something independently like people. In short, it is to let the machine find some laws from a large number of sample data through algorithms and then identify new samples or make certain predictions for the future.

The goal of training the computer in supervised learning is for it to construct a one-to-one model from input to output. During training, each machine output will be compared to the right output that has been created ahead of time and changed accordingly [28]. For example, if we want the computer to recognise the photographs of various fruits, we must train it using a huge number of human annotated fruit images. Unsupervised learning has no guide, so there is only the process of inputting data, not the process of outputting comparison. The goal of the training machine is to analyze the input data to obtain some knowledge of the data, which is typically represented by clustering. Reinforcement learning is a special kind of machine learning algorithm. In some applications, the machine needs to output a sequence of actions rather than a single result. An action excluded from the sequence is meaningless [29]. Only the sequence composed of these actions can achieve the given goal; that is, strategy is more important. Therefore, there is no best action during the execution of the machine. If the action can finally achieve the goal, that is, it is an integral part of a strategy; then, the action is good. In this case, the machine should be able to evaluate the quality of the strategy and get tips from the good action sequence learned before, so as to select the strategy with a higher success rate [30]. At present, there are many network frameworks based on the deep learning algorithms, but they are mostly based on the following four basic network frameworks.

In general, the emergence of deep learning has raised the status of machine learning to a new level, attracted extensive attention from people from all walks of life, and also led to the technological revolution in other fields. The rapid development of deep learning benefits not only from the rapid improvement of computer computing power but also from the contribution of past theories and algorithms. Although there are some limitations, such as the need for a large number of data training, good underlying hardware support, and long training time, its ability to deal with nonlinear problems and strong self-learning ability is unmatched by other algorithms.

## 3. Design of Application Model

### 3.1. Classical Feature Extraction Network

The region proposal network (RPN) region generation network utilised in the fast recurrent-convolutional neural network (R-CNN) develops the target proposal box for the location confidence problem and then approaches the target box using the boundary box regression method. The RPN network is used to judge whether the region corresponding to each point contains the required target. If so, the anchor box is used as an alternative box in the box regression and class regression layer for further correction and judgment. The method is to use a sliding window to select the region through the features to make the effective acceptance domain of the target larger and then further extract the features to perform the parallel operation of box and class in the full connection layer. Solve the problem of different scales under the same characteristics, and divide the width and height of the anchor frame by the coordinate difference to obtain a consistent prediction. The mathematical expression of the loss function is as follows:

(1) $$\begin{array}{c} \text{Loss}=\overset{N}{\underset{i}{\sum }}\left|t_{*}^{i}-W_{*}^{T}\Phi_{S}\left(A^{i}\right)\right|. \end{array}$$

In order to minimize the loss, there is a need to be calculated with the following formula:

(2) $$\begin{array}{c} W_{*}=\underset{W_{*}}{\text{argmin}}\overset{N}{\underset{i}{\sum }}\left|t_{*}^{i}-W_{*}^{T}\Phi_{S}\left(A^{i}\right)\right|+\lambda ||W_{*}||. \end{array}$$

*W*_∗_ can be obtained by applying gradient descent method or least square method. In order to prevent the over fitting phenomenon in the training process, the penalty factor is added to make the model tend to be stable. The difference between the anchor box and the confidence box is small, and the following expression is satisfied.

(3) $$\begin{array}{c} t_{w}=\log\frac{B_{w}^{gt}}{A_{w}}=\log\frac{B_{w}^{gt}+A_{w}-A_{w}}{A_{w}}=\log\left(1+\frac{B_{w}^{gt}-A_{w}}{A_{w}}\right). \end{array}$$

When the threshold is introduced, because the overlap rate between the anchor frame and the confidence frame is high, it can be regarded as an approximate linear transformation. Therefore, the desired region proposal frame can be obtained through the training of the model. While considering the use of IoU value to evaluate the distance between the prediction box and truth box, it is necessary to consider the problem that the gradient is zero and cannot be trained in the process of backpropagation when the IoU value is zero because the two boxes do not intersect. IoU can be expressed by the following formula:

(4) $$\begin{array}{c} \text{IoU}=\frac{\left|B^{p}\cap B^{gt}\right|}{\left|B^{p}\cup B^{gt}\right|}. \end{array}$$

While considering the use of IoU value to evaluate the distance between the prediction box and truth box, it is necessary to consider the problem that the gradient is zero and cannot be trained in the process of backpropagation when the IoU value is zero because the two boxes do not intersect. IoU can be expressed by the following formula. The schematic diagram of the classical feature extraction network is shown in Figure 4.

Specifically, the candidate target frame with the largest score is removed from the candidate queue and added to the second detection result queue, and then the other prediction frames in the candidate queue are compared with it. The frame with IOU greater than the threshold will be removed from the candidate queue; that is, the prediction frames with lower scores will be suppressed. Rep this process until the candidate box queue is empty and all candidate boxes in this cycle have been completed. The scores of prediction frames under different scales will be obtained in the next cycle due to the change in the anchor frame scale.

### 3.2. Improved Depth Neural Network

For real-time V detection, this chapter provides a closed center distance intersection and union ratio approach. The algorithm combines the standardized distance between the minimum closed box formed by the union of the prediction box and the target box and the center point of the target box and then integrates it into the boundary box regression calculation. The network structure diagram is shown in Figure 5.

The receptive field of deep convolution is large, so it contains more high-level semantic information. It is mainly used to detect large targets at this stage; that is, when the proportion of USV in the image is large, this stage will be dominant. Since each scale will be predicted according to the three preset anchor boxes, the corresponding center point positioning confidence loss can be expressed by the following formula:

(5) $$\begin{array}{c} {\text{Loss}}_{\text{coord}}=\lambda_{\text{coord}}\overset{S^{2}}{\underset{i=0}{\sum }}\;\overset{B}{\underset{j=0}{\sum }}\;L_{ij}^{\text{obj}}\left[{\left(x_{i}-{\overset{\wedge }{x}}_{i}\right)}^{2}+{\left(y_{i}-{\overset{\wedge }{y}}_{i}\right)}^{2}\right]. \end{array}$$

The prediction of the confidence of the prediction frame is constrained by the following formula:

(6) $$\begin{array}{c} {\text{Loss}}_{\text{conf}}=\overset{S^{2}}{\underset{i=0}{\sum }}\;\overset{B}{\underset{j=0}{\sum }}\;L_{ij}^{\text{obj}}{\left(C_{i}-{\overset{\wedge }{C}}_{i}\right)}^{2}+\lambda_{\text{noobj}}\overset{S^{2}}{\underset{i=0}{\sum }}\;\overset{B}{\underset{j=0}{\sum }}\;L_{ij}^{\text{noobj}}{\left(C_{i}-{\overset{\wedge }{C}}_{i}\right)}^{2}. \end{array}$$

That is, the network model is trained end-to-end including the confidence error of the object, the classification error of the prediction target category, and the positioning error of the prediction frame. In the process of backpropagation, the gradient will not decline or fail to reach the local optimal solution. The most direct result is that the expected training model is not obtained. Therefore, in order to make full use of the influence of loss function, some improvements are made according to the characteristics of the spatial target and prediction frame. The calculation formula of the intersection area is as follows:

(7) $$\begin{array}{c} J=\left(\min\left(x_{2},x_{2}^{gt}\right)-\max\left(x_{1},x_{1}^{gt}\right)\right)\times \left(\min\left(y_{2},y_{2}^{gt}\right)-\max\left(y_{1},y_{1}^{gt}\right)\right). \end{array}$$

The L1 loss can solve the gradient explosion problem caused by abnormally large loss value caused by outliers in the boundary box regression problem. That is, the introduction of L1 loss suppresses the influence of outliers and outliers. L1 loss is expressed as follows:

(8) $$\begin{array}{c} {\text{Smooth}}_{L_{1}}\left(x\right)=\left\{\begin{array}{c} 0.5x^{2},\;\text{ if }\left|x\right|<1,\\ \left|x\right|-0.5,\;\text{otherwise}. \end{array}\right. \end{array}$$

For the loss, the binary cross-entropy is introduced to update the predicted mask.

(9) $$\begin{array}{c} L_{\text{mask}}=\text{BCE}\left(M,M_{gt}\right)=-\left(M_{gt}\cdot \log\left(M\right)+\left(1-M_{gt}\right)\cdot \log\left(1-M\right)\right). \end{array}$$

In this way, by setting the proportion of each loss in the total loss, we can determine the branch of network key training.

## 4. Experiments and Results

The author conducted a questionnaire survey, interview, and reading test to collect data and understand the students' reading levels and reading attitudes before the experiment. After adhering to the English newspaper teaching, in order to verify the auxiliary of English newspaper reading teaching to the development of students' reading ability, the authors conducted a series of investigations in the post-test stage. The questionnaire of the posttest survey is still conducted in an anonymous way, and the questionnaires are valid. The purpose of the questionnaire survey in the posttest is to investigate students' attitudes and feelings towards the implementation of newspaper reading. The authors compare and analyze the survey results of the same questions in the pretest questionnaire and the posttest questionnaire. The survey of students' reading interests is shown in Table 1 and Figure 6.

The number of students interested in English reading has increased dramatically, with 30 percent and 46.70 percent of students indicating interest in English reading, respectively, a 33.30 percent increase over the total before the trial. The survey results show that during the experiment of English newspaper reading assisted reading teaching, most students' reading attitudes and emotions have changed positively, which proves that English newspaper reading can help students improve their reading interest. The self-assessment questionnaire for students' reading levels is shown in Table 2 and Figure 7.

It can be seen that before the experiment, only 33.30% of the students thought their reading level was high, but after the experiment, the number of students who thought their reading level was highly doubled, and the number of students who thought their reading level was high also increased by 10%, but there were still more students who thought their reading level was average, 36.70%. The survey results show that English newspaper reading, as an auxiliary reading, can make a considerable number of students increase their self-confidence, but the improvement of their level and the establishment of personal self-confidence are still subject to individual differences because it is a long and difficult process to greatly improve the self-awareness and reading level of all students. In other words, most students like the mixed learning effect evaluation index system, because the evaluation index system meets the needs of learners for the evaluation effect of English reading learning. The survey of students' weekly reading time is shown in Table 3 and Figure 8.

It can be seen that the students' reading time per week before the experiment is limited, and more than half of the students cannot guarantee even one hour per week. In the process of the experiment, the authors formulated a more detailed reading plan for students, which ensured the increase of students' reading time as a whole, and gradually made it become students' reading habits. The survey results show that almost all students can have at least one hour of reading time per week. Maintaining such a stable reading time is very important for students to improve their reading ability, which also shows that the experiment helps students develop good reading habits. Through the comparison of the results of the two questionnaires before and after, the authors find that English newspaper reading has a significant positive impact on students' English learning habits, reading ability, and reading interest, so that students have a more positive learning emotional attitude and obtain more and more comprehensive schema accumulation, which fully reflects the views of theory and schema theory, and the teaching effect is worthy of affirmation.

## 5. Conclusion

This study proves that English newspaper reading plays an auxiliary role in English reading teaching and has a positive impact on the improvement of students' reading ability through theoretical research, actual newspaper reading teaching, and experimental analysis of the development of students' reading ability. Newspaper reading improves students' interest in learning English, which is reflected not only in reading newspapers but also in other English teaching time. The authors also feel that they are more confident in their English level, show a greater desire to improve their English learning performance, and have a great sense of achievement in the expansion of their vocabulary. To increase the amount of reading is to enrich various schemata in students' minds. Anyone with English teaching experience or English learning experience knows that reading is the cornerstone of cultivating writing ability. This paper analyzes and studies the role of English newspaper reading in college English teaching, puts forward an effective analysis method of English newspaper reading teaching based on deep learning from the perspective of online and offline hybrid teaching, and verifies the effectiveness of the model through experiments.

In the process of English learning, there is no doubt about the importance of reading learning. As a result, our teachers should reflect on and investigate ways to improve their English reading teaching performance. Although this study demonstrates that English newspaper reading is beneficial to English reading instruction, it is apparent that the research has certain shortcomings. The authors hope that in the future teaching, we can also carry out empirical research on the auxiliary effect of English newspaper reading on English writing teaching, have the opportunity to exchange experience, and share achievements related to English newspaper reading teaching with teachers in other schools and further apply the research conclusions to practice for the benefit of students.

## Figures and Tables

**Figure 1:** The significance and function of English newspaper reading.

**Figure 2:** The concept of online and offline hybrid teaching.

**Figure 3:** The five characteristics of English reading teaching.

**Figure 4:** The schematic diagram of the classical feature extraction network.

**Figure 5:** The network structure diagram.

**Figure 6:** The survey of students' reading interest.

**Figure 7:** The self-assessment questionnaire for students' reading level.

**Figure 8:** The survey of students' weekly reading time.

**Table 1:** The survey of students' reading interest.

	Really like	Like	Neutral	Dislike
Before experiment	16.70%	26.70%	33.30%	23.30%
After experiment	30%	46.70%	13.30%	10%

**Table 2:** The self-assessment questionnaire for students' reading level.

	Very high	High	Neutral	Low
Before experiment	10%	23.30%	43.30%	23.30%
After experiment	20%	33.30%	36.70%	10%

**Table 3:** The survey of students' weekly reading time.

	More than 2 hours	More than 1 hour	Within 1 hour	No reading
Before experiment	10%	23.30%	43.30%	23.30%
After experiment	20%	33.30%	36.70%	10%

## Data Availability

The datasets used during the current study are available from the corresponding author on reasonable request.
